# Clinicopathological Significance of STAT3 and p-STAT3 among 91 Patients with Adenocarcinoma of the Esophagogastric Junction

**DOI:** 10.1155/2022/9311684

**Published:** 2022-10-03

**Authors:** Rui-Jie Ma, Qi-Ming Zheng, Nan Zhang, Zhi-Gang Sun

**Affiliations:** ^1^Department of Thoracic Surgery, Jinan Central Hospital, Shandong University, Jinan 250013, China; ^2^Department of Breast Disease Center, Jinan Central Hospital, Shandong University, Jinan 250013, China; ^3^Department of Thoracic Surgery, Central Hospital Affiliated to Shandong First Medical University, Jinan 250013, China

## Abstract

Adenocarcinoma of the esophagogastric junction (AEG) has increased rapidly worldwide during the last few decades. The purpose of this study is to investigate the clinical and prognostic characteristics of signal transduction and activator of transcription factor 3(STAT3) and phosphorylated STAT3 (p-STAT3) expression in AEG patients. We retrospectively analyzed the immunohistochemical results of 61 AEG patients and followed up for 5 years, while Western blot was performed on tissues from another 30 AEG patients. The results showed that STAT3 and p-STAT3 were overexpressed in AEG tissues (*P* < 0.05, *P* < 0.01). The high expression of STAT3 was significantly associated with the pTNM stage (*P* < 0.05), and the increased expression of p-STAT3 was significantly associated with depth of invasion (pT), lymph node metastasis (pN), and pTNM stage (*P* < 0.05, *P* < 0.05, *P* < 0.05). The 5-year survival rate for AEG patients was 41.0% and was significantly associated with tumor differentiation, pN, pTNM, and p-STAT3 (*P* < 0.05, *P* < 0.01, *P* < 0.05, *P* < 0.01). Cox regression analysis confirmed that tumor differentiation, pN, and high expression of p-STAT3 were independent risk factors for the 5-year survival rate in patients with AEG (*P* < 0.05, *P* < 0.01, *P* < 0.05). Our study showed that STAT3 and p-STAT3 play a critical role in AEG development.

## 1. Introduction

Adenocarcinoma of the esophagogastric junction (AEG) was first described by Siewert and Stein in 1998, defined as tumors which have their center within five centimeters of the anatomical cardia [1]. AEG is divided into three types according to the tumor's origin and location: distal esophageal adenocarcinoma, cardiac cancer, and proximal gastric cancer. The incidence of AEG has increased rapidly worldwide during the last few decades [2–4]. Obesity [5, 6] and smoking [6, 7] are independent risk factors of AEG. Most experts believe that AEG should be treated differently from gastric cancer and esophageal cancer, and multimodal treatment with surgical resection is considered the primary AEG treatment option [8]. Because of the high recurrence rate caused by invasion and metastasis, the prognosis of AEG patients is poor [9]. The TNM staging cannot adequately depict cancer prognosis because the survival rates of patients with the same TNM stage may be significantly different [10]. Therefore, it is essential to find a reliable biomarker to distinguish AEG patients with poor prognosis.

As a member of the signal transduction and activator of transcription factors (STAT) family, STAT3 is widely recognized as an oncogene. STAT3 can be activated by the Janus kinase after responding to cytokines like IL-6 [11], producing phosphorylated STAT3 (p-STAT3). p-STAT3 can enter the nucleus and increase the expression of downstream target genes like Bcl-xL, Cyclin D1, and vascular endothelial growth factor (VEGF) [12]. Recent studies show that STAT3 may serve as a critical oncogenic factor and is associated with tumor cell proliferation, invasion, migration, therapy resistance, and poor prognosis in certain types of cancer [13, 14]. The constitutive activation of STAT3 protein has been implicated in several types of malignant tumors such as esophageal squamous cell carcinoma (ESCC) [15], colorectal cancer [16], lung cancer [17], and gastric cancer [18]. However, little is known about the expression and prognostic relevance of STAT3 protein and p-STAT3 protein in AEG.

In this study, we determined the expressions of STAT3 and p-STAT3 proteins in AEG tissues and analyzed their correlations with clinicopathological parameters, including gender, age, and pTNM. Additionally, we assessed the influence of STAT3 and p-STAT3 expression on the overall survival of patients with AEG.

## 2. Materials and Methods

### 2.1. Patients and Tissue Specimens

All patients enrolled in this study underwent AEG radical surgery at the Department of Thoracic Surgery and General Surgery, Jinan Central Hospital. The specimens for immunohistochemistry staining were obtained from 61 AEG patients between January 2010 and December 2012 (Table 1), and specimens used for Western blot were obtained from 30 patients between January 2013 and June 2014 (Table 2). The inclusion criteria were as follows: (1) patients underwent complete surgery, and postsurgical pathology confirmed AEG; (2) the diagnosis of TNM stage was based on the International Union Against Cancer (2009) guideline; (3) patients accepted no preoperative chemotherapy or radiotherapy treatment before surgery; (4) patients applied comprehensive examination and multidepartment consultation before surgery to confirm they had no severe surgical contraindications that might affect prognosis. Informed consent has been obtained from all individuals included in this study. The research related to human use has complied with all relevant national regulations and institutional policies and is in accordance with the tenets of the Helsinki Declaration and has been approved by the author's institutional review board or equivalent committee.

### 2.2. Immunohistochemistry Staining

Immunohistochemistry staining for STAT3, p-STAT3 protein was detected by the streptavidin peroxidase method (SP method). AEG specimens and 10 paracancer normal tissues were fixed in 10% neutral buffered formalin and cut into 4 mm-thick slices. The analysis was applied using rabbit antibody against human STAT3 (Spring Bioscience, USA) and rabbit antibody against human p-STAT3 (Santa Cruz Biotechnology, USA) and visualized by the Envision System (Dako, Denmark). The immunohistochemistry process was described previously [16, 17]. The intensity of staining was scored as follows: negative (score 0), bordering (score 1), weak (score 2), moderate (score 3), and strong (score 4). The extent of staining was scored according to the percentage of positively stained tumor cells in the field: 0-10% (score 0), 11%-29% (score 1), 30%-49% (score 2), 50%-74% (score 3), and 75%-100% (score 4). The above two fractions multiply, and the results are divided into high expression (scores 6-12) and low expression (scores 0-5).

### 2.3. Hematoxylin–Eosin (HE) Staining

We use HE staining to confirm the pathological type and measure the degree of differentiation of tumor tissues. AEG tissues and paracancer normal tissues were fixed in 10% neutral buffered formalin and cut into 4 mm-thick slices. HE staining were prepared by using the standard method.

### 2.4. Western Blot

The fresh AEG tissues were lysed by RIPA (Biocolor Bioscience, China) with protease inhibitors and centrifuged at 12,000 rpm for 10 min at 4°C. The concentrations of protein were analyzed by BCA protein assay kit (Biocolor Bioscience, China). Equal amounts of protein were separated by 10% SDS-PAGE and transferred to PVDF membranes (Millipore, France). The membranes were blocked with 5% skim milk and incubated with primary antibodies against STAT3 (Spring Bioscience, USA) or p-STAT3 (Santa Cruz, USA), at 4°C overnight, followed by incubation with HRP-conjugated secondary antibodies (Santa Cruz, USA) for 1 h at room temperature. We used ECL reagents (Millipore, France) to visualize immunoblotted proteins, and the signals were detected by Alphamager 2200 imaging system (Alphamager, USA) and Image J analysis software (National Institutes of Health, USA).

### 2.5. Follow-Up

We ensured all 61 patients underwent AEG radical surgery between January 2010 and December 2012 came to the hospital regularly for comprehensive examination and received a complete follow-up. Overall, 32 cases received postsurgical chemotherapy, 3 cases received postsurgical radiotherapy, and 19 received both postsurgical radiotherapy and chemotherapy. Patients who died of tumors were enrolled in the prognostic analysis, and the reason for death was confirmed by the detailed preoperative evaluation and postoperative follow-up.

### 2.6. Statistical Analysis

Enumeration data were analyzed by *χ*^2^ test, Fisher's exact probability test, or *t*′ test. Univariate analysis was applied by modeling Kaplan–Meier survival curves. The log-rank test was performed to calculate the survival rate. Multivariate analysis was carried using the Cox proportional hazard model. All statistical data were analyzed using SPSS (version 13; SPSS, Inc., Chicago, IL, USA). *P* < 0.05 was considered to indicate a statistically significant difference.

## 3. Results

### 3.1. STAT3 and p-STAT3 Were Overexpressed in AEG

The results of immunohistochemistry staining shows STAT3 protein-positive signals are located in the cytoplasm and nucleus, while p-STAT3 protein-positive signals only exist in the nucleus (Figures 1 and 2). HE staining confirmed the pathological type and the degree of differentiation of AEG tumor (Figure 3). Among 61 AEG specimens detected by immunohistochemistry staining, 48 (78.7%) had high expression of STAT3, and 37 (60.7%) had high expression of p-STAT3. In 10 paracancer normal gastric/esophageal tissues, 4 (40.0%) had high expression of STAT3, and 1 (10.0%) had high expression of p-STAT3. The results of Fisher's exact probability test showed that the expression of STAT3 and p-STAT3 in AEG tissues was significantly higher than that in paracancer, normal gastric/esophageal tissues (*P* < 0.05, *P* < 0.01). The results of Western blot were analyzed by *t*′ test. The expressions of STAT3 and p-STAT3 in AEG tissues were significantly higher than those in normal paracancer gastric/esophageal tissues (STAT3: 0.6953 ± 0.17015 vs. 0.3030 ± 0.11576, *P* < 0.05; p-STAT3: 0.6000 ± 0.20978 vs. 0.1710 ± 0.07608, *P* < 0.01, Figure 4).

### 3.2. Correlation between STAT3/p-STAT3 Expression and Clinical Features of AEG

The result of immunohistochemical detection shows that the expression of STAT3 was significantly correlated with pTNM stage (*P* < 0.05, Table 1, Figure 5), but not with gender, age, tumor differentiation, pT, and pN. The expression of p-STAT3 protein closely correlated with the aggravation of pT, pN, and pTNM stage (*P* < 0.05, *P* < 0.01, *P* < 0.01, Table 1, Figure 5). No significant correlation between the expression of p-STAT3 and the gender, age, or tumor differentiation of AEG patients. In the results of Western blot, the high expression of STAT3 in AEG was positively correlated with pTNM stage (pI+pII: 0.5009 ± 0.10397, pIII: 0.8079 ± 0.6451, *P* < 0.05, Table 2, Figure 6), but no significant correlation was found between STAT3 and gender, age, tumor differentiation, depth of invasion (pT), or lymph node metastasis (pN). The level of p-STAT3 in AEG was significantly correlated with the degree of pT (pT1+pT2: 0.5071 ± 0.23776, pT3+pT4: 0.6813 ± 0.14486, *P* < 0.05), lymph node metastasis (negative: 0.4509 ± 0.24050, positive: 0.6745 ± 0.14908, *P* < 0.05), and pTNM stage (pI+pII: 0.4372 ± 0.23265, pIII: 0.6942 ± 0.12353, *P* < 0.05Table 2, Figure 6). No significantly correlation was found between the expression of p-STAT3 and gender, age, or tumor differentiation.

### 3.3. Correlation between Clinical Features of AEG Patients and 5-Year Survival Rate

The 5-year survival rate of 61 patients with AEG was 41.0% (Table 3, Figure 7). Kaplan-Meier univariate analysis showed that tumor differentiation, pN, pTNM, and p-STAT3 were related factors affecting the 5-year survival rate of AEG patients (*P* < 0.05, *P* < 0.01, *P* < 0.05, *P* < 0.01, Table 3, Figure 7). Gender, age, pT, pTNM stage, tumor location, STAT3 expression, radiotherapy, and chemotherapy were not related to the 5-year survival rate. Cox regression analysis confirmed that tumor differentiation, pN, and high expression of p-STAT3 were independent risk factors for the 5-year survival rate in patients with AEG (*P* < 0.05, *P* < 0.01, *P* < 0.05, Table 4), and postoperative treatment has no significant relationship with prognosis.

## 4. Discussion

As a member of the STAT family, STAT3 is considered the main mediator of tumorigenesis and plays an important role in the proliferation, invasion, and angiogenesis of tumor cells [19]. Constitutive activated STAT3 has been found in various cancers, including ESCC [15], colorectal cancer [16], lung cancer [17], and gastric cancer [18]. However, there is a lack of research on the mechanism and prognostic characteristics of STAT3 in AEG. The pathological type of AEG belongs to adenocarcinoma, the same as most gastric cancers, while the epidemiological characteristics and clinical symptoms are consistent with ESCC. In the research of Tian et al., STAT3 is required for the growth of ESCC cells both in vitro and in patient-derived xenografts mice [20]. In the further research of Zhao et al., the expression of STAT3 was significantly increased in ESCC and was correlated with overall survival and disease-free survival, which was an independent prognostic factor for ESCC [15]. Another research from Zhang et al. confirmed that the five-year survival rate of ESCC patients was significantly correlated with the expression of p-STAT3 [21]. A large number of studies on gastric cancer have obtained similar results. In a study of 63 patients with gastric cancer by Pan et al., STAT3 promoted the progression of TNM staging and led to a poor prognosis [22]. Besides, Wu et al. found that IL-6 secreted by cancer-associated fibroblasts can activate STAT3 signaling pathway for epithelial-mesenchymal transition and metastasis of gastric cancer in vitro and in vivo [23].

A total of 91 AEG patients were enrolled in this study. Immunohistochemical staining and Western blot were used to detect the expression of STAT3 and p-STAT3. STAT3 protein-positive signals are located in the cytoplasm and nucleus, while p-STAT3 protein-positive signals only exist in the nucleus. Compared with paracancer normal tissues, the expression of STAT3 and p-STAT3 in AEG tissues was upregulated. The level of STAT3 and p-STAT3 protein increased significantly with the aggravation of the pT and pTNM stage. We use the combination of univariate analysis and multivariate analysis to determine the prognostic factors and make the results more objective. In this study, the 5-year survival rate of AEG patients was 41.0%. Kaplan-Meier univariate analysis showed that tumor differentiation, pN, pTNM, and p-STAT3 were the related factors affecting the 5-year survival rate of AEG patients. Gender, age, pT, pTNM stage, tumor location, STAT3 expression, radiotherapy, and chemotherapy were not related to the 5-year survival rate. Cox regression analysis confirmed that tumor differentiation, pN, and high expression of p-STAT3 were independent risk factors for the 5-year survival rate in patients with AEG. Taken together, these findings suggest that the activation of STAT3 can be used as a biomarker of the poor prognosis of AEG. The results of related studies on other cancers are similar to ours. Pan et al. [22] studied the role of STAT3 in gastric cancer by immunohistochemistry, Western blot, and RT-PCR. The results showed that STAT3 was distributed in the nucleus and cytoplasm of gastric cancer, while p-STAT3 was only distributed in the nucleus. STAT3 and p-STAT3 are significantly increased in gastric cancer tissues, which affect the prognosis of patients by regulating the transcriptional activity of downstream factors EZH2. In ESCC, the distribution of STAT3 and p-STAT3 is consistent with that of gastric cancer and AEG and promotes the malignant progression of ESCC by increasing the expression of VEGF and CyclinD1 [21]. Similarly, high expression of STAT3 was found in the nucleus of endometrioid adenocarcinoma [24], high expression of p-STAT3 was found in the nucleus of hepatocellular carcinoma [25], and high expression of STAT3 and p-STAT3 was found in the cytoplasm and nucleus of breast cancer [26].

In previous studies, many genes have been confirmed to have a high expression in AEG tissues and lead to the progression of AEG tumors. VEGF is a downstream gene of STAT3, which promotes cancer growth and angiogenesis [27, 28]. In the study of Gray et al. [29], 61 AEG patients were recruited for immunocytochemical analysis of VEGF and its two receptors: VEGF-R1 and VEGF-R2. The result shows VEGF, VEGF-R1, and VEGF-R2 were overexpressed in AEG epithelial cells. Our previous study further confirmed VEGF is significantly associated with pT and pN in AEG patients [30]. Meanwhile, matrix metalloproteinase-2 (MMP-2), another downstream oncogene of STAT3 [31], is also overexpressed in AEG patients and significantly associated with tumor differentiation and pT [30]. Not only the downstream molecules but also the upstream molecules of STAT3 are highly expressed in AEG patients. IL-6 is the activator of canonical STAT3 signaling pathway which can phosphorylate JAK to activate STAT3 [32]. Besides, IL-8 [33, 34], TNF-*α* [35], and midkine [36] have also been found to be the upstream molecular of STAT3. In the research from Krzystek-Korpacka et al. [37], circulating IL-6, IL-8, TNF-*α*, and midkine were upregulated in AEG patients, and IL-6 and IL-8 participated in the cachexia of AEG. Since we have proved the role of STAT3 in AEG patients, it is valuable to find the relationship between STAT3 with its related genes in AEG.

This is the first study on the clinical and prognostic features of STAT3 in AEG. We ensured that all patients successfully underwent radical surgery and regional lymph node dissection. These tumors did not invade other organs, and routine histological examination confirmed no residual cancer cells on both sides of the cutting edge to ensure complete resection. However, there are still some limitations in this study. First of all, patients' willingness and economic status may lead patients to give up postoperative radiotherapy and chemotherapy, thus affecting the prognosis of patients. To find out whether different postsurgery therapy affects the prognosis of patients, we applied univariate analysis and multivariate analysis for the relevant data. The univariate analysis shows that neither chemotherapy nor radiotherapy has a significant correlation with the 5-year survival of patients (*P* = 0.807, *P* = 0.965), and multivariate analysis shows the same results (*P* = 0.777, *P* = 0.707). The best way to apply postoperative treatment to improve the prognosis of AEG patients reminds to be explored. Secondly, the sample size enrolled in this study is relatively small. Besides, whether the level of STAT3 and p-STAT3 would change in the different AEG subtypes is worthy for further research, and a randomized controlled prospective study with a large sample size will be considered.

## 5. Conclusion

STAT3 and p-STAT3 are highly expressed in AEG tissue. The level of STAT3 was significantly correlated with the pTNM stage, while the expression of p-STAT3 was significantly associated with the pT, pN, and pTNM stages. Tumor differentiation, pN, and high expression of p-STAT3 are independent risk factors for 5-year survival in patients with AEG. Collectively, our findings suggest that STAT3 and p-STAT3 might serve as essential biomarkers for the prognosis of AEG patients.

## Figures and Tables

**Figure 1:** Immunohistochemical staining of AEG tissue sections demonstrating STAT3 (original magnification ×400). (a) AEG tissue with high expression of STAT3. (b) AEG tissue with low expression of STAT3. (c) The paracancer normal esophageal tissue with no STAT3 expression. (d) The paracancer normal esophageal tissue with low STAT3 expression.

**Figure 2:** Immunohistochemical staining of tissue sections demonstrating p-STAT3 (original magnification ×400). (a) AEG tissue with high expression of p-STAT3. (b) AEG tissue with low expression of p-STAT3. (c) The paracancer normal gastric tissue with no p-STAT3 expression. (d) The paracancer normal esophageal tissue with no p-STAT3 expression.

**Figure 3:** HE staining of AEG tissues and paracancer normal tissues. (a) Low differentiated AEG tissue (original magnification ×40). (b) Low differentiated AEG tissue (original magnification ×200). (c) Middle differentiated AEG tissue (original magnification ×40). (d) Middle differentiated AEG tissue (original magnification ×200). (e) Paracancer normal gastric tissue (original magnification ×40). (f) Paracancer normal gastric tissue (original magnification ×200). (g) Paracancer normal esophageal tissue (original magnification ×40). (h) Paracancer normal esophageal tissue (original magnification ×200).

**Figure 4:** Western blot detection of STAT3 and p-STAT3 in AEG tissues and paracancer normal tissues. (1) Cancer tissue of AEG patients in pIII stage. (2-3) Cancer tissue of AEG patients in pII stage. (4) Cancer tissue of AEG patients in pI stage. (5) Paracancer normal tissues.

**Figure 5:** Results of immunohistochemical staining for the correlation between STAT3/p-STAT3 expressions and clinical features of AEG. (a) Correlation between STAT3/p-STAT3 expressions with gender. (b) Correlation between STAT3/p-STAT3 expressions with age. (c) Correlation between STAT3/p-STAT3 expressions with tumor differentiation. (d) Correlation between STAT3/p-STAT3 expressions with pT. (e) Correlation between STAT3/p-STAT3 expressions with pN. (f) Correlation between STAT3/p-STAT3 expressions with pTNM.

**Figure 6:** Results of western blot for the correlation between STAT3/p-STAT3 expressions and clinical features of AEG. (a) Correlation between STAT3/p-STAT3 expressions with gender. (b) Correlation between STAT3/p-STAT3 expressions with age. (c) Correlation between STAT3/p-STAT3 expressions with tumor differentiation. (d) Correlation between STAT3/p-STAT3 expressions with pT. (e) Correlation between STAT3/p-STAT3 expressions with pN. (f) Correlation between STAT3/p-STAT3 expressions with pTNM.

**Figure 7:** Survival curves of AEG patients. (a) The Kaplan-Meier's survival curve of 61 cases of AEG patients. (b) Survival curves of AEG patients with tumor differentiation. (c) Survival curves of AEG patients with negative or positive pN. (d) Survival curves of AEG patients with different pTNM. (e) Survival curves of AEG patients with low or high expression of p-STAT3 expression.

**Table 1:** Immunohistochemical staining for the correlation between STAT3/p-STAT3 expression and clinical features of AEG.

Clinical features	Patients (*N* = 61)	STAT3 expression			p-STAT3 expression		
		(−)	(+)	*P*	(−)	(+)	*P*
		13	48		24	37	
*Gender*				^∗^0.156			^∗^0.763
Male	46	12	34		19	27	
Female	15	1	14		5	10	
*Age (year)*				^∗^1.000			0.601
≥60	38	8	30		16	22	
<60	23	5	18		8	15	
*Differentiation*				^∗^0.757			1
High+medium	27	5	22		11	16	
Low	34	8	26		13	21	
*pT*				^∗^0.069			^∗^0.01
pT1+ pT2	28	9	19		16	12	
pT3+ pT4	33	4	29		8	25	
*pN*				^∗^0.117			^∗^0.001
−	25	8	17		16	9	
+	36	5	31		8	28	
*pTNM*				^∗^0.027			^∗^0.004
pI + pII	34	11	23		19	15	
pIII	27	2	25		5	22	

*P*: *χ*^2^ test, ^∗^Fisher's exact test; STAT3: signal transduction and activators of transcription factor 3; p-STAT3: phosphorylated signal transduction and activators of transcription factor 3; AEG: adenocarcinoma of the esophagogastric junction; pT: tumor invasion; pN: lymph node metastasis; pTNM: tumor stage.

**Table 2:** Western blot detection for the correlation between STAT3/p-STAT3 expression and clinical features of AEG.

Clinical features	Patients (*N* = 30)	STAT3			p-STAT3		
		STAT3 expression	*t*, *t*′	*P*	p-STAT3 expression	*t*, *t*′	*P*
*Gender*			0.032	0.198		0.256	0.884
Male	24	0.6958 ± 0.17879			0.6050 ± 0.2 1399		
Female	6	0.6933 ± 0.14445			0.5800 ± 0.20976		
*Age*			0.996	0.114		0.611	0.156
≥60	23	0.6783 ± 0.17693			0.5869 ± 0.22007		
<60	7	0.7514 ± 0.14265			0.6429 ± 0.17979		
*Differentiation*			2.508	0.091		-1.25	0.184
High+medium	10	0.5940 ± 0.19369			0.5329 ± 0.24089		
Low	20	0.7460 ± 0.13531			0.6335 ± 0.19008		
*pT*			-1.624	0.226		-2.458	0.011
pT1+ pT2	14	0.6429 ± 0.17617			0.5071 ± 0.23776		
pT3+ pT4	16	0.7413 ± 0.15573			0.6813 ± 0.14486		
*pN*			-8.278	0.225		-3.146	0.04
−	10	0.4960 ± 0.10824			0.4509 ± 0.24050		
+	20	0.7950 ± 0.08526			0.6745 ± 0.14908		
*pTNM*			-10.023	0.044		-3.974	0.01
pI + pII	11	0.5009 ± 0.10397			0.4372 ± 0.23265		
pIII	19	0.8079 ± 0.6451			0.6942 ± 0.12353		

*P*: *t* or *t*′ test; AEG: adenocarcinoma of the esophagogastric junction; STAT3: signal transduction and activators of transcription factor 3; pT: tumor invasion; pN: lymph node metastasis; pTNM: tumor stage.

**Table 3:** Univariate analysis with respect to the 5-year survival of the patients with AEG.

Clinical features	Patients	5-year survival (%)		
	61	Patients	Rate (%)	*P*
		25	41.0	
*Gender*				0.487
Male	46	18	39.1	
Female	15	7	46.7	
*Age(year)*				0.717
<60	23	9	39.1	
≥60	38	16	42.1	
*Differentiation*				0.028
Well+ moderately	27	15	55.6	
Poorly	34	10	29.4	
*pT*				0.410
pT1+ pT2	28	13	46.4	
pT3	33	12	36.4	
*pN*				0.001
−	25	17	68.0	
+	36	8	22.2	
*pTNM*				0.048
pI+ pII	34	18	52.9	
pIII	27	7	25.9	
*Chemotherapy*				0.807
No	18	8	44.4	
Yes	43	17	39.5	
*Radiotherapy*				0.965
No	46	19	41.3	
Yes	15	6	40.0	
*STAT3*				0.168
Low	13	7	53.8	
High	48	18	37.5	
*p-STAT3*				0.001
Low	24	16	66.7	
High	37	9	24.3	

*P*: log-rank test; AEG: adenocarcinoma of the esophagogastric junction; STAT3: signal transduction and activators of transcription factor 3; p-STAT3: phosphorylated signal transduction and activators of transcription factor 3; pT: tumor invasion; pN: lymph node metastasis; pTNM: tumor stage.

**Table 4:** Results of cox regression multivariate 5-year survival analysis of the patients with AEG.

Clinical features	*B*	SE	Wald	*P*	HR	95.0% CI for HR
Gender	-0.675	0.437	2.387	0.122	0.509	0.216~1.199
Age	0.280	0.372	0.567	0.451	1.323	0.638~2.743
Differentiation	1.035	0.411	6.338	0.012	2.814	1.258~6.296
pT	0.544	0.450	1.459	0.227	1.722	0.713~4.161
pN	1.851	0.598	9.566	0.002	6.366	1.970~20.572
pTNM	-0.979	0.535	3.351	0.067	0.376	0.132~1.072
Chemotherapy	-0.121	0.427	0.080	0.777	0.886	0.384~2.046
Radiotherapy	-0.160	0.427	0.141	0.707	0.852	0.369~1.967
STAT3	0.188	0.620	0.092	0.762	1.207	0.358~4.071
p-STAT3	1.314	0.563	5.448	0.020	3.722	1.234~11.223

*B*: regression coefficient; SE: standard error; Wald: Wald value; HR: hazard ratio; CI: confidence interval; AEG: adenocarcinoma of the esophagogastric junction; pT: tumor invasion; pN: lymph node metastasis, pTNM: tumor stage; STAT3: signal transduction and activators of transcription factor 3; p-STAT3: phosphorylated signal transduction and activators of transcription factor 3.

## Data Availability

The data used to support the findings of this study are included in the article.
